RETRACTED

# Application of Doctor-Nurse-Patient Co-Decision-Making Nursing Intervention Based on Evidence-Based Problems in the Rehabilitation of Acute Ankle Lateral Collateral Ligament Injury

**DOI:** 10.1155/2022/2363230

**Published:** 2022-08-19

**Authors:** Nian Wei, Yuehui Du, Shiyu Chen

**Affiliations:** Department of Foot and Ankle Surgery, Wuhan Fourth Hospital (Wuhan Orthopedic Hospital, Puai Hospital), Wuhan, Hubei 430030, China

## Abstract

**Objective:**

The aim of this study is to study the application effects of doctor-nurse-patient co-decision-making nursing intervention based on evidence-based problems in the rehabilitation of acute ankle lateral collateral ligament injury.

**Methods:**

150 patients with acute ankle lateral collateral ligament injury who were treated in the hospital between December 2020 and December 2021 were selected, and they were divided into the routine group and the evidence-based group by the random number table method, with 75 cases in each group. The patients in the routine group received routine nursing intervention, while the patients in the evidence-based group adopted doctor-nurse-patient co-decision-making nursing intervention based on evidence-based problems, and both groups were intervened for 1 month. The rehabilitation time (swelling subsidence time, fixation removal time, and normal walking time), ankle active range of motion (dorsiflexion and plantar flexion), ankle function (ankle Kofoed score) before and after intervention, and the total incidence rate of complications (tendon injury, ankylosis, and traumatic arthritis) within 1 month of intervention were compared between the two groups of patients.

**Results:**

The swelling subsidence time, fixed removal time, and normal walking time in the evidence-based group were significantly shorter than those in the routine group (*P* < 0.05). After 1 month of intervention, the ranges of motion of dorsiflexion and plantar flexion and ankle Kofoed scores of the two groups were significantly higher than those before intervention, and the abovementioned indicators in the evidence-based group were significantly higher than those in the routine group (*P* < 0.05). Within 1 month of intervention, the total incidence rate of tendon injury, ankylosis, and traumatic arthritis was significantly lower in the evidence-based group than that in the routine group (*P* < 0.05).

**Conclusion:**

Nursing intervention of doctor-nurse-patient co-decision-making based on evidence-based problems in patients with acute ankle lateral collateral ligament injury can promote postoperative rehabilitation and restore the ankle function of patients.

## 1. Introduction

Ankle lateral collateral ligament injury is one of the common soft tissue injuries, usually caused by sudden varus force of acute sprain, and the degree of lateral collateral ligament injury is related to the magnitude of varus force [1]. Improper rehabilitation of acute lateral collateral ligament injury of the ankle joint will lead to ligament relaxation, which will affect the patient's subsequent activities such as walking, running, and squatting. Routine nursing intervention in the rehabilitation of patients with acute lateral collateral ligament injury of the ankle joint is due to the lack of individualized nursing intervention for patients with different rehabilitation conditions and the difficulty in setting the rehabilitation training plan to meet the needs of the patients, resulting in an unsatisfactory rehabilitation effect, which will prolong the acute lateral ankle joint ligament injury. However, the duration of ligament injury is closely related to the prognosis of patients. When the injury time is too long, patients often have poor prognosis, which easily leads to an irreversible functional damage of joints [2]. Evidence-based problem-based nursing intervention for doctors, nurses, and patients to accompany decision-making is to implement individualized rehabilitation interventions based on the clinical condition of patients, combining the ideas and suggestions of doctors, nurses, and patients, which can fit the clinical situation of patients and meet the needs of patients as much as possible. At present, evidence-based medicine has become the mainstream of development in the medical field, and its application in nursing has gradually attracted attention. In many diseases, the nursing staff are advised to carefully, clearly, and wisely combine scientific research conclusions with clinical experience and patients' wishes to obtain evidence and use it as the basis for clinical nursing decision-making in the process of planning their nursing activities. Many reports have shown that adopting such measures can effectively promote patients' rehabilitation and reduce the adverse reactions and complications during hospitalization, but it is rarely used in the rehabilitation of patients with acute lateral collateral ligament injury of the ankle joint [3]. This study analyzes the application effect of the nursing intervention based on evidence-based problem-based doctor-nurse-patient accompaniment decision-making in the rehabilitation of acute lateral collateral ligament injury of the ankle joint.

RETRACTED

## 2. Materials and Methods

### 2.1. General Information

A total of 150 patients with acute lateral collateral ligament injury of the ankle joint who were treated in our hospital from December 2020 to December 2021 were selected and divided into the routine group and the evidence-based group by the random number table method, with 75 cases in each group.

#### 2.1.1. Inclusion Criteria

The inclusion criteria were as follows: diagnosed with acute lateral collateral ligament injury of the ankle [4]; aged 15 to 60 years old; lateral ligament injury was grade I or II; all patients had unilateral injuries; and the patients and their guardians signed the informed consent.

#### 2.1.2. Exclusion Criteria

The exclusion criteria were as follows: chronic and repeated ankle sprain; lateral ligament injury ≥ grade III; ankle dysfunction caused by other injuries; history of ankle surgery; communication impairment; bilateral ankle lateral collateral ligament injury; disturbance of consciousness or mental illness; and no tumors or major organ dysfunction.

In the routine group, gender (male/female): 38/37 cases; aged 15–59 years, mean 36.76 ± 8.90 years old; affected side: 36 cases on the left side and 39 cases on the right side; the degree of ligament injury: 31 cases with grade I, 44 cases with II; educational level: 15 cases of primary school and below, 37 cases of junior high school, technical secondary school, and high school, and 23 cases of college and above.

In the evidence-based group, gender (male/female): 39/36 cases; age 17–60 years old, with an average of 37.17 ± 10.53 years old; affected side: 35 cases on the left side and 40 cases on the right side; the degree of ligament injury: 33 cases with grade I, 42 cases with II; educational level: 16 cases of primary school and below, 35 cases of junior high school, technical secondary school, and high school, and 24 cases of college and above.

There was no significant difference in general data between the two groups (*P* > 0.05), which was comparable. This study conforms to the principles of the Declaration of Helsinki.

### 2.2. Methods

The patients in the routine group with acute lateral collateral ligament injury of the ankle joint were given routine rehabilitation nursing intervention, such as health knowledge education before rehabilitation training, affected area nursing, psychological nursing, dietary guidance, complication prevention, and ankle function training guidance.

The patients in the evidence-based group implemented the nursing intervention based on the evidence-based problem of doctor-nurse-patient co-decision-making.

#### 2.2.1. Health Education

Nurses use questionnaires, questions, and answers, etc., to understand the patient's knowledge about the rehabilitation of acute lateral collateral ligament injury before starting rehabilitation training for patients with acute lateral collateral ligament injury of the ankle joint. For example, for patients who do not understand the purpose and method of rehabilitation of acute lateral collateral ligament injury of the ankle joint, nurses can use video explanations, simulation training, etc., to show patients the content of rehabilitation training and how rehabilitation training helps patients restore the active range of motion and ankle function of the ankle joint. We take the patient's rehabilitation training plan as an example, explain the rehabilitation training objectives of each stage, and emphasize to the patient that the training plan is formulated by the medical staff after a detailed assessment of the patient's condition and physical condition and will fully fit the patient's clinical situation.

RETRACTED

#### 2.2.2. Psychological Nursing

Nursing staff increase the frequency of communication with patients, deeply understand the psychological conditions and needs of patients with acute lateral collateral ligament injury, and provide targeted psychological counseling for patients with different psychological states. For patients with acute lateral collateral ligament injuries who have a negative attitude towards the effect of rehabilitation training and are worried that the ankle joint function cannot be restored, the nursing staff can take a case that has recovered well in the past and is similar to the patient's condition as an example and inform the patient that careful cooperation with rehabilitation training can achieve recovery effects.

#### 2.2.3. Rehabilitation Training Plan Formulation

Before formulating a rehabilitation training plan, medical staff need to give a comprehensive and detailed introduction to the patient with acute lateral collateral ligament injury of the ankle joint to explain their condition and the possible impact of the injury of the lateral collateral ligament of the ankle joint on their ankle joint activities. This should be combined with targeted health education to help patients understand and master the knowledge of acute lateral collateral ligament injury and rehabilitation of the ankle joint. Then, the medical staff formulate a general rehabilitation training plan and explain to the patient the purpose and adjustable range of each stage in the plan, emphasizing that the plan is to meet the patient's requirements as much as possible and encourage the patient to actively provide opinions to strive for the best rehabilitation results. For some elderly patients who find it difficult to fully understand the content of rehabilitation training, nurses can use video and other methods to introduce the purpose and training parts of each rehabilitation training action, and appropriately guide patients to practice different rehabilitation training methods, and then ask patients their own feelings. The best training method is to work out a rehabilitation training plan with the patient.

RETRACTED

#### 2.2.4. Rehabilitation Training Implementation

During the implementation of rehabilitation according to the rehabilitation training plan jointly formulated by doctors, nurses, and patients, nurses can ask patients about the training experience of the week in the early stage and whether they need to increase the training intensity or reduce the training intensity. The staff evaluates the rationality of their opinions, and reasonable opinions can be included. For some unreasonable opinions, the medical staff need to ask the patients the reasons for their opinions and euphemistically point out that their opinions are not conducive to the rehabilitation of the ankle joint of patients with acute lateral collateral ligament injury. During the implementation of the rehabilitation training plan, the medical staff try their best to meet the needs of patients and adjust the rehabilitation training plan in a targeted manner when conditions permit.

#### 2.2.5. Complication Prevention

Nursing staff inform patients of possible tendon injuries, ankle stiffness, traumatic arthritis, and other complications and related influencing factors through health education before rehabilitation training. During rehabilitation training, medical staff guide patients to avoid mistakes, training methods, correcting their behavior, and instructing patients to report to the medical staff in time when they feel uncomfortable with the training intensity, adjusting the training plan, and avoiding excessive training intensity and damage to the tendon. Both groups were treated for 1 month.

### 2.3. Observation Indicators

The observation indicators were as follows: (1) Comparison of rehabilitation time: we record and compare the time of swelling subsidence, immobilization removal, and normal walking time between the two groups of patients. (2) Comparison of the active range of motion of the ankle joint: we measure and compare the active range of motion of the ankle joint in dorsiflexion and plantar flexion before and after the intervention in the two groups [5]. Measurement of dorsiflexion: the patient remains in a sitting position, bends the knee to 90°, the ankle joint is placed in a neutral position, the protractor is placed 2.5 cm from the midpoint line of the ankle, the patient's toes are raised, and the dorsum of the foot is approaching the front of the calf to form the ankle joint, we measure the dorsiflexion angle, the normal range is 0 ∼ 25°. Determination of plantar flexion: The patient's posture is the same as the test dorsiflexion, the toes are drooping, the dorsum of the foot is far from the front of the calf, and the ankle joint is measured. The higher the range of dorsiflexion and plantar flexion, the higher the active range of motion of the ankle joint. (3) Comparison of ankle joint function: The ankle joint Kofoed score [6] was used to measure and compare the ankle joint function of the two groups of patients before and after intervention, including pain, function, and range of motion. 75< the score ≤85 was considered as good, < the score ≤75 was considered as passing, and the score ≤70 was considered as poor. The higher the score, the better the ankle function of the patient. (4) The total incidence of complications: The total incidence of tendon injury, ankle stiffness, and traumatic arthritis in the two groups of patients within 1 month of intervention was recorded and compared.

RETRACTED

### 2.4. Statistical Methods

SPSS 22.0 was used for analysis, % was count data, *χ*^2^ test was performed, and rank data were subjected to rank sum test; $\bar{x}$ ± *s* was measured data, *t* test was performed, and *P* < 0.05 was considered a significant difference.

## 3. Results

### 3.1. Comparison of Recovery Time

In the evidence-based group, the swelling subsided, the fixation was removed, and the normal walking time was significantly shorter than those in the routine group (*P* < 0.05) as shown in Table 1 and Figure 1.

### 3.2. Comparison of Active Range of Motion of the Ankle Joint

After 1 month of intervention, the dorsiflexion and plantar flexion activities of the two groups were significantly higher than those before the intervention, and the values of the evidence-based group were significantly higher than those of the routine group (*P* < 0.05) as shown in Table 2 and Figure 2.

### 3.3. Comparison of the Ankle Joint Function

One month after the intervention, the ankle Kofoed scores of the two groups were significantly higher than those before the intervention, and the values of the evidence-based group were significantly higher than those of the routine group (*P* < 0.05) as shown in Table 3.

### 3.4. Comparison of the Total Incidence of Complications

Within 1 month of intervention, the total incidence of tendon injury, ankle stiffness, and traumatic arthritis in the evidence-based group was significantly lower than that in the conventional group (*P* < 0.05) as shown in Table 4.

## 4. Discussion

Acute lateral collateral ligament injury of the ankle joint is mostly caused by a sports sprain, which affects the function and stability of the patient's ankle joint and can seriously lead to repeated ankle joint injury. Rehabilitation training is very important for patients with an acute lateral collateral ligament injury of the ankle joint, which directly affects the recovery of the patient's ankle joint [7]. Therefore, it is necessary to study the appropriate nursing intervention mode for the rehabilitation of patients with acute lateral collateral ligament injury in order to promote their ankle recovery.

RETRACTED

After conservative treatment, patients with acute lateral collateral ligament injury still need to implement rehabilitation training to restore the balance of their ankle muscles. However, conventional rehabilitation training interventions are usually implemented by medical staff after making a rehabilitation training plan. Most patients are passively trained and lack understanding of rehabilitation training conditions and activities, resulting in insufficient participation and enthusiasm for rehabilitation training, which affects the effect of rehabilitation training and increases the time required for their ankle joint to recover [8]. Evidence-based problem-based nursing intervention for doctors, nurses, and patients to accompany decision-making is a nursing intervention based on the patient's condition requirements to achieve the ideal rehabilitation effect [9]. In the results of this study, the swelling subsided, the fixation was removed, and the normal walking time of the patients in the evidence-based group was significantly shorter than those in the conventional group. After 1 month of intervention, the dorsiflexion, plantar flexion range of motion, and ankle Kofoed scores of the two groups were significantly higher than those before the intervention, and the scores of the evidence-based group were significantly higher than those of the routine group, suggesting that the joint decision-making nursing intervention of doctors, nurses, and patients based on evidence-based problems has obviously promoted the recovery degree of the ankle joint. One month after the operation is the critical period for the functional recovery of the ankle joint, and the progress of functional recovery in this period is very important for the patients in the future [10, 11]. The reason is that the nursing intervention based on evidence-based problem-based decision-making with doctors, nurses, and patients first analyzes the factors that affect the recovery time and effect of patients with acute lateral collateral ligament injury of the ankle joint and then implements the nursing intervention from the aspects of health knowledge, psychology, rehabilitation training plan, complications, etc. Nursing intervention can comprehensively reduce the risk of risk factors affecting the rehabilitation of patients with acute collateral ligament injury, mainly because when formulating and implementing the rehabilitation training plan, medical staff first conducted a questionnaire survey on patients with acute ankle collateral ligament injury to understand their lack of health knowledge and then implemented targeted health education to achieve the effect of filling the examination gap [12, 13]. Before formulating the rehabilitation training plan, we fully explain the purpose, meaning, and method of the rehabilitation training to the patient; formulate a preliminary rehabilitation training plan according to the clinical condition of the patient; introduce the reasons for the training to the patient in detail; encourage the patient to express their own ideas and propose plan revision suggestions; and jointly formulate a rehabilitation training plan with patients, which can improve the patient's participation and subjective initiative, so that the rehabilitation training plan can be carried out smoothly, ensure its application effect, and promote the recovery of the patient's ankle joint [14, 15].

RETRACTED

In the rehabilitation process of patients with acute collateral ligament injury of the ankle joint, some patients suffer from complications such as improper rehabilitation training intensity, ankle stiffness, and traumatic arthritis, which affect the ankle joint recovery effect and daily living function [16]. In routine rehabilitation training, because the training plan is formulated by medical staff and there is a lack of communication with patients, it is easy to cause the rehabilitation training plan to fail to meet the needs of patients and there is an insufficient participation of patients, which affects their enthusiasm and cooperation and increases the risk of complications. In the results of this study, within 1 month of intervention, the total incidence of tendon injury, ankle stiffness, and traumatic arthritis in the evidence-based group were significantly lower than that in the conventional group, indicating that the evidence-based problem-based medical-nursing-patient accompanying decision-making nursing intervention for acute rehabilitation of patients with lateral collateral ligament injuries of the ankle can reduce the risk of complications. The reason is that the nursing intervention model based on evidence-based problems can be patient-centered, fully adapt to the clinical situation of patients, and implement targeted nursing interventions from health knowledge, psychology, complications, etc., and rehabilitation training plans. We ask patients for their thoughts and opinions when formulating to improve patient participation, thus increasing patients' enthusiasm and cooperation for rehabilitation training. This can effectively avoid the occurrence of improper training intensity in the process of rehabilitation training and reduce the risk of complications such as tendon injury, ankle stiffness, and traumatic arthritis [17, 18].

RETRACTED

In conclusion, nursing intervention based on evidence-based problem-based decision-making with nursing intervention for patients with acute lateral collateral ligament injury of the ankle joint can reduce the risk of complications, shorten the rehabilitation time, and help restore the active range of motion of the ankle joint and ankle joint function. It can be used as one of the clinical nursing intervention programs.

## Figures and Tables

**Figure 1:** Rehabilitation time of the two groups of patients.

**Figure 2:** Active range of motion of ankle joint before and after intervention in the two groups of patients.

**Table 1:** Comparison of recovery time between the two groups of patients (*n* = 75, *d*, $\bar{x}$ ± *s*).

Group	Swelling subsided	Fixation removal	Normal walking
Evidence-based group (*n* = 75)	8.16 ± 1.74	17.09 ± 4.51	41.69 ± 5.37
Regular group (*n* = 75)	9.15 ± 2.11	18.88 ± 4.51	44.29 ± 5.90
*T*	3.124	2.424	2.822
*P*	0.002	0.017	0.005

**Table 2:** Comparison of active ankle range of motion before and after intervention in the two groups of patients (*n* = 75, °, $\bar{x}$ ± *s*).

Group	Time	Dorsiflexion	Plantar flexion
*Evidence-based group*	Before intervention	6.25 ± 1.00	18.65 ± 3.24
	After intervention	17.97 ± 3.07^a^	39.27 ± 2.97^a^

*Regular group*	Before intervention	6.48 ± 0.96	18.13 ± 3.09
	After intervention	16.33 ± 2.69^a^	37.89 ± 3.76^a^

*T* after intervention		3.480	2.677

*P* After intervention		0.001	0.008

Compared with the group of before intervention, ^*a*^*P* < 0.05.

**Table 3:** Comparison of ankle joint function before and after intervention in the two groups (*n* = 75, cases, %).

Group	Time	First rate	Well	Qualified	Poor
*Evidence-based group*	Before intervention	0 (0.00)	3 (4.00)	21 (28.00)	51 (68.00)
	After intervention	20 (26.67)^a^	34 (45.33)^a^	18 (24.00)^a^	3 (4.00)^a^

*Routine group*	Before intervention	0 (0.00)	5 (6.67)	23 (30.67)	47 (62.66)
	After intervention	11 (14.67)^a^	25 (33.33)^a^	31 (41.33)^a^	8 (10.67)^a^

*Z* after intervention		3.033			

*P* after intervention		0.002			

Compared with the group of before intervention, ^*a*^*P* < 0.05.

**Table 4:** Comparison of the total incidence of complications between the two groups of patients during the intervention period (*n* = 75, cases, %).

Group	Tendon injury	Ankle stiffness	Traumatic arthritis	Total incidence
Evidence-based group	3 (4.00)	2 (2.67)	1 (1.33)	6 (8.00)
Routine group	9 (12.00)	4 (5.33)	3 (4.00)	16 (21.33)
*χ * ^*2*^	3.261	0.174	0.257	5.327
*P*	0.071	0.677	0.612	0.021

RETRACTED

## Data Availability

The raw data supporting the conclusion of this article will be available from the authors without undue reservation.
